# *In vitro* and *In vivo* study targeting the development of Unani Antidermatophytic Cream: Implication of Herbal Formulations in Treatment of Dermatophytosis

**DOI:** 10.1016/j.heliyon.2023.e16154

**Published:** 2023-05-09

**Authors:** Hina Anjum, Ghulamuddin Sofi, Moyad Shahwan, Mohd Shahnawaz Khan, Anas Shamsi, Shariq Shamsi

**Affiliations:** a Dept. of Ilmul Saidla (Unani Pharmacy), National Institute of Unani Medicine, Bangalore, India; b Dept. of Ilmul Advia (Unani Pharmacology), National Institute of Unani Medicine, Bangalore, India; c Center of Medical and Bio-Allied Health Sciences Research (CMBHSR), Ajman University, Ajman, P.O. Box 346, United Arab Emirates; d Department of Clinical Sciences, College of Pharmacy and Health Sciences, Ajman University, Ajman, P.O. Box 346, United Arab Emirates; e Department of Biochemistry, College of Sciences, King Saud University, Riyadh, 11451, Saudi Arabia; f Centre of Medical and Bio-allied Health Sciences Research, Ajman University, United Arab Emirates

**Keywords:** Chrysophanol, Dermatophytosis, Dermal irritation, Ringworm, Water removable base

## Abstract

*Panwad* (Ca*ssia tora* L.), *Sarshaf* (Brassica nigra L.) and *Kunjad* (*Sesamum indicum* L.) have been used in the treatment of ringworm infection since ancient times and are documented in classical literature of Unani Medicine. These plant drugs give promising results when used topically in the form of paste (*zimad*). Hence, the development and evaluation of a cream containing extracts of *Tukhm-e-Panwad (Cassia tora* L*.), Sarshaf (Brassica nigra* L*.),* and *Kunjad (Sesamum indicum* L*.)* was carried out to get better efficacy of the drugs. A total of 16 batches (F1–F16) of cream were prepared by adding varying concentrations of hydro-alcoholic extract of the drugs (20%, 40% and 50%) in water removable bases, and three batches were selected as final batches (F4-20%, F6-40% and F16-50%). *In vitro* antidermatophytic activity was conducted to optimize MIC against dermatophytosis-causing fungi. Dermal irritation of the prepared cream was determined in New Zealand Albino Rabbits. *In vivo* testing of the different concentrations of the prepared cream (20%, 40%, and 50%) was also carried out using Wistar rats to assess the antidermatophytic activity. Final batches showed good results in all the tested parameters and significant *in vitro* and *in vivo* antifungal activity in a dose-dependent manner. No microbial growth was seen in the prepared formulation. The study revealed significant antidermatophytic activity of the prepared cream against dermatophytosis-causing fungi. Hence, it can be concluded that the prepared cream can be an alternative topical agent with safe and effective antifungal activity for treating dermatophytosis.

## 1 Introduction

The most common skin infection includes fungal infections, mainly affecting the stratum corneum layer of the skin but may also affect the deeper layer of the skin. Among various types of fungal infection, dermatophytosis is most commonly found, which is also known as tinea, depending upon the site or location of the lesion [[1], [2], [3]]. Dermatophytosis is a group of fungal infections commonly caused due to the three types of fungal genera: *Trichophyton, Microsporum, and Epidermophyton* [[4], [5], [6]]. The lesions are characterized by one or more circular, sharply circumscribed, slightly erythematous, dry, scaly, and usually hypopigmented patches. Progressive central clearing produces annular outlines that give them the name “ringworm” [2].

The management of dermatophytosis involves treatment by oral and topical antifungal agents in the conventional system of medicine [7]. However, increased episodes of recurrent infection and growing resistance to these antifungal agents, and a typical presentation of the dermatophytic lesion have mandated the development of a novel formulation for the treatment.

Traditional medicine has played an essential role in providing treatment for various diseases. *Qooba* is one of the skin diseases described in the Unani System of Medicine (USM). It resembles dermatophytosis in symptoms such as scaly, dry circular lesions associated with slight oozing and intense itching. USM has many drugs which have significant results in treating *Qooba*/Dermatophytosis. One such compound formulation recommended for dermatophytosis is mentioned in classical literature, consisting of *Panwad (Cassia tora* L.*), Sarshaf (Brassica nigra* L*.),* and *Kunjad (Sesamum indicum* L.*)* [8]. *Panwad (Cassia tora* L.*)* is a known antifungal plant because of an anthraquinone, chrysophanol, which inhibits the cell wall synthesis and leads to the delayed sporulation of fungus, and reduces spore germination [9]. These three drugs are recommended to be applied in the form of paste [8] prepared by mixing the powder of crude drugs and water. Using these drugs in the form of paste is difficult. It shows lesser bioavailability due to the lesser duration of contact between medicine and diseased part as the paste scraps off the skin easily. Though this preparation has some disadvantages, it has been used by Unani physicians for decades because of its efficacy, even in this presently available form. Therefore, considering the formulation's efficacy, our study aimed to modify the formulation (paste) into a newer one, which would be more acceptable to patients and more beneficial to treat dermatophytosis. This study was carried out by taking the extract of the same ingredients as mentioned in *Tibb-e-Ahsani, i.e., Tukhm-e-Panwad, Sarshaf, Kunjad,* and modified into a novel dosage form that was formulated as per the modern pharmaceutics and comparatively more acceptable by the patients, i.e., Cream.

Various excipients were used depending on the property they impart to the semisolid topical preparation. Standardizing the newly formulated cream is imperative to provide valid data for quality control. So, a physicochemical evaluation of the cream was also done. Only optimizing, formulating, and developing a cream would not solve our objective because the ultimate aim of any medicine/dosage form is to treat the patients. Therefore, it was necessary to check the efficacy of every formulation. So, *in vitro, irritancy, and in vivo studies were* also done to confirm the efficacy of the cream.

## 2 Materials and methods

### 2.1 Materials

All the excipients and chemicals used in the preparation of cream were procured from Bengaluru, India. Ethanol for extract preparation was purchased from Coatings and Coating Pvt. Ltd. Mumbai (Maharashtra). .

### 2.2 Procurement and identification of herbal drugs

The ingredients of the formulation were procured from Bengaluru. Ingredients were identified and authenticated by Senior Botanist, Assistant Prof. S. Noorunnisa Begum, Centre for Repository of Medicinal Resources (C-RMR), *Trans*-Disciplinary University (TDU), Attur, Bengaluru. The voucher specimens (*Cassia tora* L. - 5240*, Brassica nigra* L. - 5241*, Sesamum indicum* L. - 5242) have been deposited in the museum of the Institute of *Trans*-Disciplinary Health Sciences and Technology, Bengaluru.

### 2.3 Test organisms

*Trichophyton mentagrophytes* (MTCC-7687) fungal strain was used in the study. The strain was purchased from Microbial Type Culture Collection and Gene Bank (MTCC), CSIR- Institute of Microbial Technology, Chandigarh. It was obtained in freeze-dried form and was subcultured on Potato Dextrose agar. The strain was preserved at Dextrose Technologies Pvt. Ltd. Bangalore. Fungal spore suspension was taken for the study.

### 2.4 Commercial topical antifungal agent

Fluconazole cream (0.5%) and Clotrimazole cream IP 1% were obtained from local drug retail outlets in Bangalore. These commercial topical drugs were used as a standard control for *in vitro* and *in vivo* antidermatophytic activity.

### 2.5 Preparation of extracts

The foreign & earthy matter and residual materials were removed from all the ingredients. After that, all the ingredients were coarsely powdered separately with the help of an electric grinder and pulverizer. Each coarsely powdered drug was then subjected to the extraction separately with water & ethanol in the ratio of 1:1 using a soxhlet extractor. The extract was filtered and then concentrated to dryness on a water bath.

### 2.6 Preparation of cream batches

Sixteen batches of the cream (F1–F16) were prepared using water removable/miscible bases [[10], [11], [12]] by fusion method [13,14]. The cream's low, moderate, and high concentration (w/w) was prepared by incorporating the extract (20%, 40%, and 50%) and other excipients of the formulation in varying concentration. (Table 1).

**Table 1:** Composition of different formulation batches (% w/w).

S.No.	Ingredients	F1	F2	F3	F4	F5	F6	F7	F8	F9	F10	F11	F12	F13	F14	F15	F16
a.	Stearic acid	14%	10%	10%	10%	10%	10%	10%	10%	10%	10%	10%	10%	10%	10%	10%	10%
b.	Cetyl alcohol	1.0%	2.0%	3.0%	3.0%	3.0%	4.0%	3.0%	4.0%	3.0%	3.0%	2.0%	2.0%	2.0%	3.0%	2.0%	3.0%
c.	Span 60	2.0%	2.0%	2.0%	2.0%	2.0%	2.0%	2.0%	2.0%	2.0%	2.0%	2.0%	3.0%	3.0%	2.0%	2.0%	2.0%
d.	Coconut oil	1.0%	3.0%	3.0%	3.0%	3.0%	3.0%	3.0%	3.0%	3.0%	3.0%	3.0%	–	3.0%	3.0%	3.0%	3.0%
e.	Tween 60	2.0%	1.5%	1.5%	1.5%	1.5%	1.5%	1.5%	1.5%	1.5%	1.5%	1.5%	3.0%	1.5%	1.5%	1.5%	1.5%
f.	Menthol	–	–	–	–	–	–	–	–	–	–	–	–	–	1.0%	1.0%	–
g.	Sorbitol 70% liquid	3.0%	5%	3.0%	3.0%	3.0%	3.0%	3.0%	3.0%	3.0%	3.0%	3.0%	3.0%	3.0%	2.0%	2.0%	2.0%
h.	Propylene glycol	–	10%	7.0%	10%	10%	6.0%	10%	6.0%	8.0%	10%	12%	10%	10%	8.0%	8.0%	8.0%
i.	Micro crystalline cellulose	–	–	–	–	–	–	–	–	–	–	–	–	40%	–	–	–
j.	Methyl paraben	0.1%	0.1%	0.1%	0.1%	0.1%	0.15	0.1%	0.1%	0.1%	0.1%	0.1%	0.1%	0.1%	0.1%	0.1%	0.1%
k.	Propyl paraben	0.05%	0.05%	0.05%	0.05%	0.05%	0.05%	0.05%	0.05%	0.05%	0.05%	0.05%	0.05%	0.05%	0.05%	0.05%	0.05%
l.	Extract	20%	20%	20%	20%	40%	40%	60%	60%	60%	60%	60%	60%	60%	60%	60%	50%
m.	Distilled water	q.s	q.s.	q.s.	q.s.	q.s.	q.s.	q.s.	q.s.	q.s.	q.s	q.s.	q.s.	q.s.	q.s.	q.s.	q.s.

### 2.7 Evaluation of cream

All sixteen batches were evaluated on their organoleptic properties: appearance, odour, colour, texture, homogeneity, thermal cycle, phase separation, etc., and pH value. Based on these parameters, F4 (20%), F6 (40%), and F16 (50%) were selected as final batches. These three final batches were further evaluated for viscosity, spreadability, extrudability, rancidity, stability, microbial load, and phytochemical screening. Chromatographic analysis and *In vitro* evaluation were also performed using the highest concentration batch (F16-50%). The dermal irritation of the prepared cream was done using the F16-50% batch, whereas *in vivo* antidermatophytic activity was determined in all three final batches, i.e., F4, F6, and F16.

#### 2.7.1 Organoleptic properties

The prepared formulation cream was inspected visually for its physical appearance, colour, odour, texture, phase separation, and homogeneity. Except for homogeneity and texture, all the characteristics were inspected visually; however, the homogeneity and texture were tested by pressing a small quantity of the formulated product between the thumb and index finger. The consistency of the formulation and the presence of coarse particles were used to evaluate the texture and homogeneity of the formulation. Immediate skin feel (stiffness, grittiness, and greasiness) was also assessed [15].

#### 2.7.2 Oily feel

Oily feel was checked by spreading the cream on the skin's surface and washing it with tap water.

#### 2.7.3 Thermal cycle test

The portion was stored at 5 °C for 48 h and then at 25 °C for 48 h. The procedure was repeated 3 times, and their stability and appearance were evaluated [15].

#### 2.7.4 After feel

Emolliency, slipperiness, and amount of residue left after applying the fixed amount of cream were checked [16].

#### 2.7.5 Type of smear

After applying cream, the type of film or smear formed on the skin was checked [16].

#### 2.7.6 Removal

The ease of removing the cream was examined by washing the applied part with tap water [16].

#### 2.7.7 Determination of pH

The pH measurement of each formulation was done in triplicate as per the method described by Gemeda et al. and Pal et al. [15,16].

#### 2.7.8 Determination of viscosity

The viscosity of the prepared cream was determined by using a Capillary viscometer.

#### 2.7.9 Determination of spreadability

Mutimer et al. apparatus was used to determine the spreadability [11,16].

#### 2.7.10 Determination of extrudability

The prepared cream was filled in a collapsible tube container. The extrudability was determined in terms of the weight of cream required to extrude 0.5 cm of ribbon of cream in 10 s [11]**.**

#### 2.7.11 Rancidity test

Rancidity was determined by the method given in Unani Pharmacopoeia of India [17].

#### 2.7.12 Stability studies

The prepared cream was packed in collapsible aluminium tubes and subjected to stability studies at three different temperatures viz., 5 °C, 25 ^°^C, and 40 °C for a period of 3 months. Samples were withdrawn at 15-day time intervals and evaluated for physical appearance and pH [18].

#### 2.7.13 Phytochemical screening of the cream

The prepared cream was subjected to phytochemical screening per the standard procedures to reveal the presence of various active phytoconstituents like saponins, tannins, alkaloids, anthraquinone, glycosides, sugars, proteins, and phenols [19].

#### 2.7.14 Microbial contamination

The formulated cream with the highest concentration of extract (F16-50%) was assessed for total microbial load [[20], [21], [22]].

### 2.8 Qualitative analysis by GC-MS (gas chromatography-mass spectrometry)

The cream analysis with the highest extract concentration (F16-50%) was done by gas chromatography [23,24].

### 2.9 Experimental procedures

#### 2.9.1 *In vitro* antifungal assay

##### 2.9.1.1 Determination of zone of inhibition

The antimicrobial efficacy of the cream (F16-50%) was tested by a well-diffusion method. Wells of 6 mm diameter were punched on plates containing specified agar media. 100 μl of fungal spore suspension was spread onto the agar plates. The wells were then loaded with varying concentrations of the cream (20, 30, 40, 50, 60, 70, 80, and 90 mg/ml). Fluconazole (0.5%) was used as a positive control. Fungal plates were incubated at room temperature for 3–5 days. The diameter of zone of inhibition for cream was measured [[25], [26], [27], [28]].

##### 2.9.1.2 Determination of minimum inhibitory concentration (MIC)

The MIC value was determined by using the agar dilution method. The fungal isolate (*Trichophyton mentagrophyte*) was grown on PDA and incubated at room temperature. The fungal spore suspension was prepared. The fungal spores were suspended in sterile 0.9% saline, and the turbidity of the suspension was measured and adjusted using a spectrophotometer at 530 nm to a final transmission ranging from 75%. This has resulted in fungal spore suspension of approximately 1 × 10^5^ to 5 × 10^5^ CFU/ml. The inoculum quantitation was performed by using quantitative colony plate counts of the cell suspension to obtain the actual number of CFU per millilitre. The adjusted suspension was vortexed and diluted 1:100 in distilled water. The diluted suspension was vortexed, and 0.01-ml aliquots (using a calibrated quantitative loop) were spread onto Potato dextrose agar plates with a glass spreader. The plates were incubated at room temperature, and the CFU per millilitre counts were determined when growth was evident [[25], [26], [27], [28]].

#### 2.9.2 *In vivo* study

##### 2.9.2.1 Ethical statement

The experimental protocol comprised dermal irritation of the prepared cream on New Zealand albino rabbits and its *anti*-dermatophytic activity on Wistar rats.

Experimental trials involving animals were authorized by the Government of India under registration no. 953/GO/Re/S/06/CPCSEA issued by the Committee assigned for the Purpose of Control and Supervision of Experiments on Animals (CPCSEA) and validated by the Institutional Animal Ethics Committee, National Institute of Unani Medicine, Bangalore, India for this work (IAEC/7/16/IS/07).

##### 2.9.2.2 Skin irritation test

The degree of dermal irritation of the prepared cream (F16-50%) was determined in New Zealand Albino rabbits using the semi-occluded dermal irritation test method [29].

Three healthy young adult albino rabbits weighing about 1.0 kg–1.5 kg were used as per the Organization for Economic Co-operation and Development guideline 404 (OECD 404) for the acute dermal irritation test. As per the OECD guidelines, dermal irritation was performed initially using one animal. Approximately 24 h before the test, fur was removed by trimming the dorsal area of the trunk of the animal, followed by shaving the fur by using a razor in an area of approximately 6 cm^2^ [29]

A dose of 0.5 gm of the prepared cream was applied to a small area (approximately 4 cm^2^) of skin and covered with a gauze patch held in place with non-irritating tape. The patch was loosely held in contact with the skin using a suitable semi-occlusive dressing for 4 h. At the end of the exposure period, i.e., 4 h, the residual substance was removed using normal saline without altering the existing response or integrity of the epidermis [30].

After the initial test, the prepared cream was found to be non-irritant. Hence, the confirmatory test was carried out using two additional animals, each with one patch, for an exposure period of 4 h.

All three animals were examined for any signs of erythema and edema. For the initial test in one animal, the test site was examined immediately after the patch was removed. Dermal reactions were graded and recorded according to the grades given in OECD guidelines 404.

The primary irritation index (PII) was calculated by dividing the sum of erythema and edema scores of the grading intervals by the number of grading intervals. The formulation was then classified using PII scoring method [29,31].

(1) $$PII=\sum \frac{Erythema\;and\;edema\;grades\;at\;0,24,48,72\;hrs}{Number\;of\;observations}$$

##### 2.9.2.3 *In vivo* antidermatophytic activity

• **Preparation of dermatophyte inocula**

*In vivo* antidermatophytic activity was carried out using different concentrations of prepared cream i.e. 20%, 40% and 50% (F4, F6 and F16). *Trichophyton mentagrophytes* MTCC 7687 was selected as it is the commonest type of fungus causing dermatophytosis [32]. To prepare the fungal inoculum to be injected into the rats, several petridishes of Potato Dextrose Agar (PDA, Dextrose Technologies Pvt. Ltd.) were seeded with T. mentagrophytes and incubated at 30 °C for 7 days. The colonies were scrapped from the plates with a sterile cell scrapper and added in normal saline (0.9%). This cell suspension was prepared fresh and used to challenge animals [33].

• **Dermal infection of animals**

Both male and female Wistar rats (130-200 gms) were used for the study. The animals were divided into five groups-group 1- negative control; Group 2- standard control; Group 3, Group 4 and Group 5 were test groups for 20%, 40% and 50% of the prepared cream (Table 2). Using scissors, an area of about 6 cm^2^ on the dorsal flank of each rat was trimmed, followed by close shave of the area using a razor. After 24 h of the shaving of fur, 125 μl of a suspension of *T. mentagrophytes* spores (spore count 1 × 10^6^) was applied to a surface of about 4 cm^2^ area within the shaved zone, which was previously abraded by using medium grit sandpaper. Evidence of infection was revealed by direct observation of the infected area, followed by agar culture of scrapings from the area and microscopic observation of the resulting fungi from the scrapping [31,33].

• **Treatment of infected animals**

Animals were treated by dermal application of the test formulation, which started on 3rd day after the animal infection and was continued daily (each morning). All animals were infected and treated except those of group 1 [31,32].

• **Clinical surveillance of the treatment**

The clinical evaluation was done every 7th day during a period of 21 days, i.e. on 7th, 14th and 21st day of the treatment. Clinical response was monitored by assigning a score between 0 and 4 to each infection site: 0 (no inflammation); 1 (for flaking skin with mild inflammation); 2 (for slight lesions with moderate inflammation); 3 (for moderate lesions with severe inflammation) and 4 (for severe inflammation plus crust formation). These scores were used to compare the efficacy of different treatment groups. The following equation estimated percent efficacy (Equation (2)):

(2) $$Percent\;efficacy=100-\left(T\times \frac{100}{C}\right)$$

where T = total score of treatment arm; C = total score of untreated control.

The total score for any group denoted the average clinical score from the animals in the same group [31,33].

### 2.10 Statistical analysis

Data on irritation are presented as visual scores based on the irritation scale as per OECD 404 of erythema and edema grading system, and PII was calculated, whereas the inhibition diameters of cream preparation were expressed in mm. ANOVA one-way test was employed to analyze the data obtained from separate groups on various analysis days. p < 0.05 was considered significant.

The experimental setup is depicted in Table 2.

**Table 2:** Experimental design.

S. No.	Grouping	Treatment given	No. of animal	Route of drug administration
**1.**	Group 1 (Negative control)	No treatment	6	-0-
**2.**	Group 2 (Standard control)	Clotrimazole cream 1%	6	Local application
**3.**	Group 3 (test group)	20% prepared cream	6	Local application
**4.**	Group 4 (test group)	40% prepared cream	6	Local application
**5.**	Group 5 (test group)	50% prepared cream	6	Local application

## 3 Results

### 3.1 Physico-chemical evaluation of the cream

The physicochemical evaluation showed better results in the final batches as compared to other batches (Table 3).

**Table 3:** Physicochemical evaluation of final batches.

Properties	F4	F6	F16
Appearance	Opaque, Smooth, Semisolid	Opaque, Smooth Semisolid	Opaque Smooth Semisolid
Colour	Dark brown	Dark brown	Dark brown
Odour	Pleasant	Pleasant	Pleasant
Consistency	Excellent	Excellent	Excellent
Homogeneity	Homogenous	Homogenous	Homogenous
Oily feel	Present	Present	Present
Grittiness	Absent	Absent	Absent
Stickiness	Absent	Absent	Absent
Absorption	Excellent	Excellent	Excellent
After feel	Emollient	Emollient	Emollient
Type of smear	Non-greasy	Non-greasy	Non-greasy
Removal	Easily removable	Easily removable	Easily removable
Phase separation	Absent	Absent	Absent
Viscosity (cP)	3.87 ± 0.014	4.029 ± 0.002	4.48 ± 0.001
Spreadability (g.cm/sec)	2.11 ± 0.040	1.30 ± 0.075	1.10 ± .005
Extrudability	Good	Good	Good
Rancidity	Negative	Negative	Negative

### 3.2 Phytochemical screening

The phytochemical screening revealed all the classes of compounds (saponins, tannins, alkaloids, anthraquinone, glycosides, sugars, proteins and phenols) in the prepared cream (Table 4).

**Table 4:** Qualitative analysis of final three batches of prepared cream (F4, F6, F16).


Phytochemical Constituents	Phytochemical test	Results
Alkaloid	Mayer's test	+ve
	Dragendorff's test	+ve
Carbohydrates	Anthrone test	+ve
	Fehling's test	+ve
	Benedict's test	+ve
Flavanoids		+ve
Glycosides	Glycosides test	+ve
Phenols	Ferric chloride test	+ve
	Lead acetate	+ve
Proteins	Millon's test	+ve
Tannins	Lead acetate test	+ve
	Ferric chloride test	+ve

### 3.3 Microbial contamination

The total microbial load was found to be nil for the prepared cream. No growth was observed in agar plates against any pathogen (Table 5).

**Table 5:** Total Microbial load.

S. No.	Test	Results
1.	Total microbial count (cfu g)	No growth
2.	Total yeast and mould count (cfu g)	No growth

### 3.4 Qualitative analysis of prepared cream

The various phytoconstituents found in this study resemble the previous studies, which provide strong evidence of authentication of the drugs and serve the purpose of quality control (Table 6, Fig. 1).

**Table 6:** Compounds detected in GC-MS analysis.

S.No.	Compounds	Molecular Formula	Molecular weight
1.	*Cis*-1,3,3trimethylbicyclo u[3.1.0]Hexane-1-Carboxaldehyde	C_10_H_16_O	152
2.	4-Allyl-2-methoxy-phenol	C_10_H_12_O_2_	164
3.	4-Tridecanol	C_13_H_28_O	200
4.	4-Pentadecanol	C_15_H_32_O	228
5.	N-methyl-*n*-(*p*-nitrophenyl)furfurylamine	C_12_H_12_O_3_N_2_	232
6.	4-Hexadecanol	C_16_H_34_O	242
7.	Methyl 5,9-hexadecadienoat	C_17_H_30_O_2_	266
8.	Silane, [(11-chloroundecyl)oxy]trimethyl-	C_14_H_31_OClSi	278
9.	9,12-Octadecadienoic acid (Z,Z)-	C_18_H_32_O_2_	280
10.	9*Z*,12*Z*-Octadecadienoic acid methyl ester (Linoleic acid methyl ester)	C_19_H_34_O_2_	294
11.	Linoleoyl chloride	C_18_H_31_ClO	298
12.	*cis*-13-Eicosenoic acid	C_20_H_38_O_2_	310
13.	Sinapine(2-[(E)-3-(4-hydroxy-3,5-dimethoxyphenyl)prop-2-enoyl]oxyethyl-trimethylazanium)	C16H24NO5+	310.37
14.	6,11-Eicosadienoic Acid, Methyl Ester	C_21_H_38_O_2_	322
15.	Fumaric acid, decyl pent-4-enyl ester	C_19_H_32_O_4_	324
16.	Erucic acid	C_22_H_42_O_2_	338
17.	2-Chloroethyl linoleate	C_20_H_35_O_2_CL	342
18.	1-Cyclopentyl Eicosane	C_25_H_5_O	350
19.	Fumaric acid, pent-4-enyl tridecyl ester	C_22_H_38_O_4_	366
20.	Fumaric acid, 3-methylbut-3-enyl tetradecyl ester	C_23_H_40_O_4_	380
21.	Fumaric acid, 3-methylbut-3-enyl pentadecyl ester	C_24_H_42_O_4_	394
22.	Fumaric acid, hexadecyl 3-methylbut-3-enyl ester	C_25_H_44_O_4_	408

**Fig. 1:** Total ION chromatography (gas chromatography).

### *3.5* *In vitro* antidermatophytic activity

The formulated cream (F16-50%) was evaluated for its *anti*-dermatophytic activity against *Trichophyton mentagrophyte* by agar well diffusion method, and the diameter of the zone of inhibition was measured. The concentrations of cream used for trial 1 showed less inhibition against the test organisms, so higher concentrations of cream were used in the trial 2 studies.

The diameter of zone of inhibition was found highest at 90 mg concentration of the cream against *Trichophyton mentagrophytes.*

Prepared cream was also compared with standard and zone of inhibition at 20 mg/ml and 50 mg/ml was measured. Zone of inhibition of standard i.e. Fluconazole 0.5% against *T. mentagrophytes* was found to be 31 mm at 20 mg/ml and 42 mm at 50 mg/ml respectively (Table 7).

**Table 7:** *Anti*-dermatophytic activity of Prepared cream.

Concentration (mg/ml)	Diameter of Zone of inhibition in mm
	Trichophyton mentagrophytes
20	0
30	0
40	0
50	0
60	10
70	20
80	17
90	26
Positive control −20 (Fluconazole)	31
Positive control −50 (Fluconazole)	42

#### 3.5.1 Minimal inhibitory concentration of highest concentration batch (F16)

MIC of the prepared cream (F16-50%) was evaluated by using Agar dilution method and was found to be 55 mg for *Trichophyton mentagrophytes.* (Table 8).

**Table 8:** Minimal inhibitory concentration of highest concentration batch F16 at 530 nm.

Concentration (mg/ml)	*Trichophyton mentagrophytes.*
5	1.876
10	1.800
15	1.655
20	1.492
25	1.200
30	0.973
35	0.712
40	0.439
45	0.200
50	0.198
55	0.000
60	0.000
65	0.000
70	0.000
75	0.000
80	0.000
85	0.000
90	0.000
Positive control (Organism without antifungal)	1.879
Positive control(with antifungal) −20 (Fluconazole)	0.000
Negative control (Media)	0.000

### 3.6 *In vivo* study

#### 3.6.1 Dermal irritation test

The degree of dermal irritation was evaluated as per OECD guidelines 404. Dermal irritation studies proved that the cream formulation at 50% extract concentration was non irritant. The primary irritation index was found to be a negligible limit of 0.01 and indicated safe for human use.

#### 3.6.2 *Anti*-dermatophytic activity

Infected Wistar rats were monitored daily for signs of infection. Initial signs such as scaling and redness of the infected area appeared by 2nd day post-infection in the infected animals. As the infection progressed for the next few days, redness intensified with the marked scaling of the lesion. Signs of inflammation were visible, along with the formation of the circular ring-like structure around the lesion. The treatment started at 72 h post-infection. From the 7th day of treatment, the lesion intensity started dropping in the treated groups in a dose-dependent manner, i.e. 20% cream had a lesser effect than 40% and 50%. Cream formulation with 50% extract concentration showed significant changes on 7th day itself. However, the prepared cream with lower and moderate concentrations of extract (F4-20% and F6-40%) gradually overcomes the infection from the 14th and 21st day of the treatment, respectively. Simultaneously, lesions continued to increase in the untreated group (negative control). Treatment with clotrimazole 1% and prepared cream with the highest concentration (F16-50%) resulted in complete healing of the infected site. Most of the signs in the skin lesion were similar to those observed in moderate forms of clinical dermatophytosis in humans (Fig. 2).

**Fig. 2:** *Anti*-dermatophytic activity of Prepared cream. (A) Animals three days after infection. (B) Prepared cream applied on lesions started on 4th day post infection. (C) 7th day, (D) 14th day and (E) 21st day post treatment with cream.

## 4 Discussion

In recent years, several antifungal agents in MSM have been introduced into clinical practice, including griseofulvin, terbinafine, itraconazole, fluconazole [7,34]. However, their spectrum of action is narrow, and many have specific adverse effects, such as gastrointestinal disturbances, nephrotoxicity, hepatotoxicity and leucopenia [31,32,35]. Treating dermatophytic infection is often long and expensive, and there have been increasing reports of antifungal resistance [31,33]. Increased incidence of fungal infections due to the rise in immunocompromised population, coupled with the resistance to antifungal and toxicity during prolonged treatment, has been the reason for an extended search for newer drugs to treat opportunistic infections. Thus, it is imperative to develop such treatment of broad spectrum dermatophytic infection with lesser adverse effects [25,31,35]. There have been a large number of plant species which shows significant antifungal activity. Unani ancient literature has mentioned numerous plants and mineral origin drugs that can be used topically or orally to treat dermatophytosis [36,37]. An important formulation for the treatment of dermatophytosis is mentioned in *Tibb-e-Ahsani*, which is recommended to be used in the form of paste [8]. It comprises of *Panwad (Cassia tora* L.*), Sarshaf (Brassica nigra* L.*),* and *Kunjad Siyah (Sesamum indicum* L*).* These single drugs are also prescribed by various Unani physicians alone for treating dermatophytosis because of various good actions like *Cassia tora* L. possess detergent and blood purifier action, which helps to clear the skin, waste products and putrefied materials from the blood [38]. *Brassica nigra* L. has been used since ancient times for its rubeficient*,* demulcent and detergent properties. The rubeficient action of this drug helps to increase the blood circulation of the part where it is applied and thereby helps to treat the disease. The demulcent action of *Sarshaf* helps to liquefy the thick and viscous matter. *Sesamum indicum* L. is used as a vehicle in many topical preparation as it possesses emollient action which provides necessary lubrication to combat excessive dryness and pruritus resulting from the deposition [[39], [40], [41], [42]].

Many recent studies have also proven these drugs' effect in treating ringworm infection. *Cassia tora* L shows antifungal activity due to chrysophanol and crysophanic acid- 9- anthrone and other anthraquinones such as emodine, physcion and rhein [43,44]. Brassica nigra L. is a valuable source of glucosinolates, polyphenols and flavonoids. On hydrolysis by the enzyme myrosinase, glucosinolates produce d-glucose isothiocynates, and nitrites. These isothiocynates inhibit spore germination and show potent antifungal activities [23]. *Sesamum indicum* L. has lecithin which shows emollient action and therefore, it is effective in dermatitis and dry skin [45]. Lignan compounds are found in higher concentrations in sesame seeds. These phenolic compounds act as an antimicrobial agent by inactivation of microbial adhesion, enzymes and other proteins, through non specific forces like hydrogen bonding, covalent bonding, hydrophobic interactions and inhibiting cell wall polymer synthesis [46].

The particular formulation selected for the study is mentioned to be used as paste, by taking an equal quantity of powdered drugs, i.e. Panwad, Sarshaf and Kunjad and making a paste by mixing with water. Although, good results of this paste, but have many problems in the pre-application and application. So making it more stable, easy to use, and efficacious an attempt has been made to modify this paste preparation into a more convenient novel dosage form cream. Creams tend to be preferred when an occlusive effect is not necessary and are frequently chosen for wet and weepy skin conditions because they are able to emulsify with the serous exudates of dermatitis [47]. Specifically, o/w cream is non-occlusive because it does not deposit a continuous film of water-impervious liquid. However, such creams can deposit lipids and other moisturizers on and into the stratum corneum and restore the tissue's hydration ability, i.e. the preparation has emollient properties [12]. The excipients used in the preparation of cream are very well suited for the purpose of target drug delivery only up to the superficial layer of the skin i.e. stratum corneum [48]. Water removable bases were used to prepare emulsion. O/W creams rub into the skin; the continuous phase evaporates and increases the concentration of a water soluble drug in the adhering film. The concentration gradient for drug across the stratum corneum therefore increases, promoting percutaneous absorption [12].

Hence, in this study, o/w emulsion was selected for the preparation of the cream. Including an emulsifying agent or agents is necessary to facilitate actual emulsification during manufacture and ensure emulsion stability during the product's shelf-life. The non-ionic surfactants tend to be less irritant and less toxic than their anionic and particularly cationic counterparts. These are not susceptible to pH change and the presence of electrolytes [[10], [11], [12]]. Hence, this study used non-ionic surfactants such as Span 60 and Tween 60 to prepare o/w emulsion.

Moreover, stearic acid is widely used as an emulsifying and solubilizing agent in topical preparations. When partially neutralized with alkalis or triethanolamine, stearic acid is used to prepare creams. The partially neutralized stearic acid forms a creamy base when mixed with 5–15 times its own weight of aqueous liquid, the appearance and plasticity of the cream being determined by the proportion of alkali used [49]. Therefore, stearic acid was used in the preparation of this cream.

Cetyl alcohol was used in cream because of its emollient, water-absorptive, and emulsifying properties. It enhances stability, improves texture, and increases consistency. The emollient properties are due to the absorption and retention of cetyl alcohol in the epidermis, where it lubricates and softens the skin while imparting a characteristic ‘velvety’ texture. In oil-in-water emulsions, cetyl alcohol improves stability by combining with the water-soluble emulsifying agent. The combined mixed emulsifier produces a close-packed, monomolecular barrier at the oil–water interface, forming a mechanical barrier against droplet coalescence [49].

Coconut oil was used to prepare cream because it forms a readily absorbable base. In addition, coconut oil has been reported to have antifungal activity against a range of *Candida* and *Trichophyton* species [[49], [50], [51]]. This activity may be beneficial for the treatment of other types of fungi [49]. Methyl and propyl paraben were used to prepare cream as antimicrobial preservatives. Propylene glycol and sorbitol were used as humectants in the formulation of cream because propylene is proven to show antidermatophytic against *Trichophyton* spp*,* which can add to the better efficacy of our formulation [52].

Total 16 batches were prepared and were designated as F1–F16. Hydroalcoholic extract was taken in different concentrations (20–60%) and different excipients with minor concentration changes. Significant *in vitro* antidermatophytic activity for *T. mentagrophytes* was shown in the prepared cream (F16-50%). The zone of inhibition was found to be 26 mm at 90 mg and be minimum inhibitory concentration was 55 mg. This shows that prepared cream would be useful for the treatment of dermatophytosis. The skin irritation test also revealed that the formulated cream is non-irritant on rabbit skin. The primary irritation index was found to be zero and indicated safe for human use.

Trichophytosis induced in rats is a well-established model for testing topical antifungal agents [53]. This model was used in this study, and the results prove that formulated cream possesses promising dose-dependent *in vivo* antifungal activity against a virulent strain of T. mentagrophytes. Formulated cream showed variable effects in different concentrations on different days of treatment, i.e. 7th, 14th and 21st days. The formulated cream produced: mild effects after seventh day of treatment only at a higher concentration (F16-50%); mild, moderate and excellent effects after the fourteen and twenty-one day of treatment at 20%, 40% and 50% concentration respectively. Hence, it shows that the formulated cream at 50% concentration was able to cure infected animals completely after twenty one days of treatment. The results also show the same effect after twenty-one days of treatment in clotrimazole. These results indicate that this formulation can be used as an alternative to clotrimazole to cure dermatophytosis.

## 5 Conclusion

This study demonstrates that the cream prepared by the extract of *Tukhm-e-Panwad* (*Cassia tora* L.), *Sarshaf* (*Brassica nigra* L.) and *Kunjad* (*Sesamum indicum* L.) possesses antidermatophytic properties without irritation effect. These results may justify using all three crude drugs in the USM to cure dermatophytosis. Moreover, various excipients such as coconut oil and propylene glycol may also contribute to the efficacy of prepared cream.

## Author contribution statement

Hina Anjum, Ghulamuddin Sofi: Performed the experiments; Analyzed and interpreted the data; Wrote the paper.

Moyad Shahwan, Mohd Shahnawaz Khan: Analysis and interpreted the data; Wrote the paper.

Anas Shamsi, Shariq Shamsi: Conceived and designed the experiments; Analyzed and interpreted the data; ; Wrote the paper.

## Data availability statement

Data included in article/supplementary material/referenced in article.

## Authors's statement

**Hina Anjum:** Performed the experiments; Analyzed and interpreted the data; Wrote the paper. **Ghulamuddin Sofi:** Performed the experiments; Analyzed and interpreted the data; Wrote the paper, Moyad Shahwan: Analyzed and interpreted the data; Wrote the paper. **Mohd Shahnawaz Khan:** , Analyzed and interpreted the data; Wrote the paper. **Anas Shamsi:** Conceived and designed the experiments; Analyzed and interpreted the data; Wrote the paper. **Shariq Shamsi:** Conceived and designed the experiments; Performed the experiments; Analyzed and interpreted the data; Wrote the paper.

## Declaration of competing interest

The authors declare that they have no known competing financial interests or personal relationships that could have appeared to influence the work reported in this paper.
